The article "Application of Infusion Control System Based on Internet of Things Technology in Joint Orthopedics Nursing Work" was retracted in 2023. Reasons: signs of a paper mill; suspected computer-generated content; unreliable results or conclusions; lack of ethics approval or compliance.

# Application of Infusion Control System Based on Internet of Things Technology in Joint Orthopedics Nursing Work

**DOI:** 10.1155/2021/6691258

**Published:** 2021-03-26

**Authors:** Xia Bai, Qiaoli Wang, Shengqin Cao

**Affiliations:** ^1^Department of Joint Surgery, The Fourth People's Hospital of Jinan, Jinan, Shandong 250031, China; ^2^Nursing Department, The Fourth People's Hospital of Jinan, Jinan, Shandong 250031, China; ^3^Department of Spinal Surgery, The Fourth People's Hospital of Jinan, Jinan, Shandong 250031, China

## Abstract

In recent years, the Internet of Things technology has flourished, and there have been corresponding practical results in various fields. In medical care, the introduction of Internet of Things technology must also be a new trend in the development of hospital informatization, and it is the development stage of the digital medical process. The traditional infusion system shows that the infusion bottle is not replaced in time, the infusion waiting time is too long, the infusion efficiency is too low, and the existing medical staff is far from meeting the needs of the huge infusion population. Therefore, this article proposes a technology based on the Internet of Things application of the infusion control system in joint orthopedics nursing work to improve the efficiency of infusion in nursing work. This article deeply learns and uses the Internet of Things technology to build a new infusion management and control system, which is applied to joint orthopedics nursing treatment. This paper designs the application research experiment of the infusion control system. Through the Internet of Things technology, the relevant data in the infusion process are uploaded and sent to the network center of the hospital. Nursing staff can directly see the infusion situation directly through the computer console. This article compares and analyzes two different infusion systems and draws conclusions. The infusion ringing rate of the control group was 81.3%, and the infusion ringing rate of the IoT group was 29.8%; the time for timely replacement of the infusion bottle after IoT data control was 13.89 min, compared to 19.76 min before. A variety of data results show that the infusion management and control system based on the Internet of Things technology has played a great role in joint orthopedics care, which can greatly improve the efficiency of infusion, replace the infusion or deal with failures in time for patients, and improve patient satisfaction.

## 1. Introduction

Injection therapy is the basic medical intervention that not only is the most widely used in hospitals but also an important way to clinical treatment and relief of patients [1]. Since 1972, the American Intravenous Influenza Disease Association has set the goal of providing patients with the highest quality, safe, and effective injections and continuously improving the quality of the injections. However, with the continuous progress of society, the demand for medicines has also increased, the types of medicines used have increased, and the average number of medicine bottles per patient has continued to increase. Now, there is a shortage of nurses in family hospitals, and the demand for patients is increasing.

In joint orthopedics nursing work, the infusion control system will maximize the use of Internet technology to solve practical problems [2], make the monitoring and management of intravenous infusion more intelligent and refined, optimize the infusion management process, and improve the quality of infusion connection. To ensure the quality of infusion treatment, the safety of nurses and improvement of work efficiency are now the most urgent management issues that should be injected into the hospital.

Nobre G C circular economy is a term that has emerged since the 1970s and has become increasingly important in the past few years, partly due to the scarcity of natural resources available in the environment and changes in consumer behavior. Cutting-edge technologies like big data and the Internet of Things (IoT) have the potential to leverage the adoption of CE concepts by organizations and society to make them more realistic in our daily lives [3]. Therefore, it is very important for researchers interested in this topic to understand the current status of ongoing research worldwide and to have an overall understanding of it. He reviewed the bibliometrics of the Scopus database from 2006 to 2015, focusing on the application of big data/Internet of Things in the CE environment. This allowed 30,557 CE documents to be combined with 32,550 unique big data/Internet of Things research, resulting in 70 matching publications, and content and social network analysis using the “R” statistical tool. Then he compared it with some current industry initiatives. However, his research lacks practical application value [4]. Dobkin B H showed that although the theory of exercise learning has led to the practice of evidence-based medicine, few trials have shown that one theoretical treatment is better than another poststroke treatment. The improvement of skills is not as clinically meaningful as people hope. He reviewed some possible explanations and then potential technical support solutions. The quality and intensity of home training can be monitored remotely via the Internet, and the quality and intensity of training can be optimized. A group of home-based rehabilitation IoT (RIoT) devices can provide a theory-driven collaborative intervention for walking, reaching, mastering, strengthening, and fitness. The RIoTs may include wearable activity recognition sensors and instrumented rehabilitation equipment [5], which are transmitted via radio to a smartphone or tablet to continuously measure the repetitiveness, speed, accuracy, strength, and temporal characteristics of movement. Using remote rehabilitation resources, the therapist will interpret the data and provide self-management behavior training through goal setting and guidance to improve compliance. However, there are too many subjective factors in the experiment process [6]. Bob Metcalf, the inventor of Ethernet and a well-known technology visionary, once said that we have built the Internet to meet the world's demand for cheap and clean information in the past 63 years. In the next 63 years, we will build Ethernet to meet the world's demand for cheap clean energy. The Internet was born out of revolutionary advancements in electronics, telecommunications, information technology, equipment, and applications. Although it was originally an Internet that connected people, in 2008, it connected more things than people. This exponential growth is mainly as the IoT. He predicts that, by 2020, the IoT will add 50 billion new connections [7]. So far, the US public power grid is an integral, weakly interconnected, and synchronized AC power grid, powered by thousands of large power plants, which are centrally monitored and controlled [8]. For various reasons, this legacy grid method proved to be impractical at present and in the future. However, his research needs to be more supplemented [9].

The innovations of this article are as follows: (1) combining qualitative research with quantitative research, fully combining research data with practical application value, and showing the practical value of this research; (2) combining theoretical research with empirical research and in-depth study based on the theoretical basis of the IoT technology combined with the actual infusion control system to conduct empirical investigations. The innovation of this paper is to emphasize the full combination of the IoT technology and the infusion management system and the feasibility exploration in the actual application process.

## 2. Application Method of Infusion Control System Based on Internet of Things Technology in Joint Orthopedics Nursing Work

### 2.1. Internet of Things Technology

The Internet of Things refers to the use of sensing devices such as radio frequency identification systems or infrared induction systems to give objects intelligence according to a certain protocol and connect objects to the Internet through ports [10], thereby forming a distributed network of interconnected objects and realizing intelligent object identification, tracking, monitoring, and management technology [3, 11]. It connects the object to the network through the information detection device according to the protocol, communicates through the media, and realizes the functions of intelligent identification, configuration, monitoring, and monitoring. Internet of Things refers to the comprehensive integration of existing terminal equipment and equipment such as sensors, mobile terminals, industrial systems, numerical control systems, household smart devices, and video surveillance systems with “intrinsic intelligence” [12]. In addition, people who transmit wireless terminals through various wireless, cable long-distance, and/or short-distance communication networks include “external activation” such as “smart objects or animals” and “smart trash,” as well as various assets such as RFID-equipped and other equipment [13]. Establish interfaces, integrate functions with cloud-based SaaS applications, and adopt appropriate information security mechanisms in the internal network environment. Perform real-time monitoring and positioning to realize task management, project management, remote control, security protection, remote maintenance, online upgrades, statistical reports, decision support, cockpit dashboards, and the integration of “high-performance management, control, and application.” Other types of management and the service functions play a role in high-security protection [14, 15].

(1) $$\begin{array}{c} \left(\text{NSID}-\text{IoT}\right)+\left(\text{NB}-\text{IoT}\right)+\left(\text{OID}-\text{IoT}\right)=\frac{\text{IOE}}{\text{IOE}*N}=\text{IoT.} \end{array}$$

Among them, NSID-IoT is the abbreviation of the IoT under the telecommunication network number, NB-IoT is the abbreviation of the cellular-based narrowband IoT, OID-IoT is the abbreviation of Xintongyunke, IOE is the abbreviation of the Internet of Everything, and these together form IoT [16].

Simply put, IoT is the transmission and control of information between objects and between people and objects. The basic technologies to realize the IoT include sensor technology, radio frequency identification technology, integrated system technology, intelligent technology, and nanotechnology [17]. As shown in Figure 1, this represents the IoT core technology diagram. Sensor technology is the core technology. It has the earliest use time and plays the most basic role. In the computer field, it needs to convert analog signals into digital signals so that computers can process them. Radiofrequency identification technology is a kind of sensor technology, which combines radiofrequency and embedded technology, and is widely used in applications in the fields of identification of objects, fingerprint recognition, and facial recognition [18]. The integrated system is a complex integrated system. Its applications can be found in every corner of life. For example, MP3 around you can also be used in aerospace technology. Simply put, it is mainly used to classify and process information. Intelligent technology relies on intelligent systems. Only intelligent systems can fully realize the purpose of communication and information transmission between objects and users. Nanotechnology is mainly used in many fields such as physics, chemistry, and biology. For a long time, we have proposed the use of good network for health care. The initial stage refers to the realization of intelligent data management based on wireless frequency identification technology and equipment through the combination of protocol communication protocols and the Internet [19]. Medical IoT is medical treatment, health management, and IoT technology applied to elderly care [20, 21].

Medical network “things” refer to healthy people, healthy people, patients, and so on, doctors, nurses, medical equipment, inspection machines, drugs, and so on, and various things related to medical service activities. The “connection” with the medical Internet of Things refers to the mutual connection and interaction of information, as well as the sharing of information [22]. The medical Internet “network” is a “network” that is organically connected to the “things,” understanding the objects of medical services, exchanging objects and objects, real-time monitoring of medical care service data, continuous monitoring and management, and correct medical and health decisions.

### 2.2. RFID Technology

RFID technology refers to frequency and identification technology. In other words, it refers to achieving the purpose of confirming the target. RFID has a wide range of uses. Typical applications include animal chips, car chips for antitheft devices, access control, parking space control, production line automation, material management, and medical management [23]. Radiofrequency identification technology uses the rapid information exchange and storage technology of radio wave information, combines wireless communication and data access technology, and connects to the database system to realize noncontact two-way communication for the purpose of identification and data exchange. In the identification system, the reading, writing, and communication of electronic tags must be performed through electromagnetic waves. According to different communication distances, it can be divided into short distance and long distance. Therefore, the data exchange method between the reading/recording device and the electronic tag is also divided into loading configuration and backscattering configuration [24, 25].

The complete RFID system includes card readers, electronic tags, so-called transponders, and application software systems [23]. The principle of the operation is that the card reader sends the energy of the radio wave of a specific frequency to the operation circuit to send internal data. Currently, the identifier will continue to receive and interpret the data and send it to the application for corresponding processing. Generally speaking, radio frequency identification technology has the characteristics of applicability, high efficiency, independence, and simplicity [26, 27]. Its reading and writing speed are extremely fast, and it can read the contents of multiple tags at the same time, shortening the information transmission time. In RFID, each tag is unique, has a one-to-one correspondence, and can be well used in logistics and transportation applications. The equipment and universality required by RFID technology are gradually popularized in everyone's smartphones [28].

(2) $$\begin{array}{c} A=\text{IDS}⊕K_{1}\;⊕\;n_{1},\\ B=\left(\text{IDS}\vee K_{2}\right)+n_{2},\\ {\bar{K}}_{1}=\text{Rot}\left(K_{1}\;⊕\;n_{2},K_{1}\right),\\ {\bar{K}}_{2}=\text{Rot}\left(K_{2}\;⊕\;n_{1},K_{2}\right),\\ C=\left(K_{1}⊕{\bar{K}}_{2}\right)+\left({\bar{K}}_{1}\;⊕\;K_{2}\right),\\ D=\left({\bar{K}}_{2}+I\;DS\right)⊕\left(\left(K_{1}\;⊕\;K_{2}\right)\vee {\bar{K}}_{1}\right). \end{array}$$

During the execution of the RFID system, perform the above formula operations in the reader to obtain D and complete the tag data exchange with the electronic device. Among them, the reader and the tag share the key K, pseudonym IDS, and the reader finds the corresponding keys K1 and K2 according to the pseudonym.

Radiofrequency identification technology can be divided into passive, active, and semiactive RFID. The classification standard is based on the power supply mode of the tag [29,30]. Passive RFID system usually requires power supply; it can achieve a short powered electromagnetic induction coil to complete the information exchange. It can achieve short-term power supply through electromagnetic induction coils to complete the information exchange process. It is generally used in information exchange places with short distances, such as bus cards and ID cards. It is characterized by small enough volume, simple structure, low production cost, long service life, and so on [31]. The development time of active RFID is not long; it needs to rely on an external power supply, mainly used in highway toll stations. It has the characteristics of long-distance transmission of information, high efficiency, and high performance. And more than the previous generation has a function to recognize multiple tags at the same time. Semiactive RFID is a compromise between passive and active RFID. First, it must be activated by external stimuli and then positioning and recognition, information acquisition, and information transmission [32].

The development of RFID technology combined with multiple fields shows the characteristics of high frequency, network, and flexibility. Combined with the medical department, the infusion control system plays an important role in joint orthopedic surgery care, and its applications are becoming more and more extensive.

### 2.3. Cloud Computing Technology

Cloud computing is a distributed computer that discards huge computer data processing programs into countless small programs through a cloud network, processes them, and analyzes designated processes through a system composed of multiple servers. Get the Applet result and return it to the user. Simply put, in the early days of cloud computing, it was a combination of simple decentralized computing, work-sharing solutions, and calculation results. Therefore, cloud computing is also called network computing. According to this technology, tens of thousands of data can be processed in a short time (several seconds) and powerful network services can be realized.

The key technology in cloud computing is that first, its architecture intact is able to create the necessary environment and conditions; the system is intelligent enough, but also for the variation signal of quick reaction capability; second, it can monitor resources, cloud system database resources are huge, and data update speed is fast. Cloud computing's resource monitoring is conducive to managing the load and usage of resources and maximizing the effectiveness of resource information; third, it can implement automated deployment operations in mass. Among the data, the resources in the database can be divided, deployed, and installed to provide users with various application services.

Cloud computing can fully implement the above three technologies in the injection management control system. Through the use of full-architecture cloud computing, resource monitoring, and automatic development technology, the injection system can be solved and the effect of joint plastic surgery treatment can be improved.

## 3. Application Experiment of Infusion Control System Based on Internet of Things Technology in Joint Orthopedics Nursing Work

### 3.1. Subject

This article chooses to use convenience sampling method to select data. The data source is Y hospital patients who underwent infusion therapy in joint orthopedics nursing from April 2016 to June 2016. According to the admission order, 210 cases were selected as the control group, and 358 cases were admitted after selection for the research object of the IoT group.

A total of 210 patients were in the control group (158 males and 52 females; 20–83 years old, average 55.3 ± 9.22 years; number of infusion bottles per day: average 7.3 ± 3.41 bottle; education level: 50 cases of junior high school and below, 73 cases of high school, and 87 cases of junior high school and above). There are 358 patients in the infusion management group of the IoT (226 males and 132 females; 19–82 years old, with an average of 54.1 ± 9.96 years; number of infusion bottles per day: 3–16, with an average of 7. 1 ± 3.53 bottle; education level: 43 cases of junior high school and below, 67 cases of high school, and 248 cases of junior high school and above). There was no statistically significant difference between the two groups of patients in terms of gender, age, number of infusion bottles, education level, and so on (*P* < 0.05).

### 3.2. Experimental Method

#### 3.2.1. Internet of Things Infusion Management Group

1. *Design Principle*. In the daily work of joint orthopedics nursing, the Internet of Things technology is used for the infusion control system, real-time monitoring procedures are adopted for the entire infusion process, the information is uploaded and transmitted in time, and the nursing team members provide real-time feedback. Through the Internet of Things technology to implement all-weather monitoring of each patient and each hospital bed to achieve a 24-hour uninterrupted effect, members of the joint orthopedics nursing team can know the patient's infusion status at any time in the nurse's station or in the mobile state. The replacement of infusion bottles and the handling of accidental infusions can improve the work efficiency of medical staff and bring patients a better experience of seeing a doctor.
2. *System Composition.* The infusion management and control system consists of infusion monitoring instruments, data receivers, and computer screens (with network interfaces), and the structure is shown in Figure 2. First, complete the collection of infusion data, including infusion time and infusion volume, through the infusion monitoring instrument; then upload the infusion-related information and send it to the data receiver. Each bed in the room is equipped with an infusion monitor, which is hung on a hook under the screen window. Each information bar is equipped with a data receiver, and the monitor will send data. The monitor will monitor various infusion parameters, such as infusion time, infusion speed, remaining infusion time, dynamic appearance of changes in the liquid level in the container, infusion failure, and reminders when the infusion is complete.

Statistically analyze the two quality groups of infusion management and the quality group related to nursing business effects. Patients in the infusion management group use an infusion monitoring system based on IoT technology. The injection package is hung on the side injection monitoring unit. After the injection time is 2 minutes, the monitoring unit automatically detects that the integrated central monitoring jet is monitoring the upper bed number, and the nurse management department will issue an alarm. The nurse can prepare the liquid in the patient's bag in advance according to the situation. After 1 minute of the remaining injection time, the system will wake up again and the nurse will change the fluid from the bed. If the injection speed changes in the middle or the injection stops due to a needle lock, an alarm signal will occur. During the injection process, there is no need to automatically analyze the information of the injection process through software.

#### 3.2.2. Control Group

This control group mainly uses regular injection processes to perform regular inspections of nurses and patients or related staff and participates in injection monitoring, injection management, and manual statistics of injection process information.

### 3.3. Observation Indicators

1. The work efficiency index of nurses compares the number of infusion-related bell ringing, the number of nurses going back and forth to the nurse station, and the average number of daily steps taken by the nurses between the two groups.
2. Compare the relevant infusion reaction indicators of the two groups of patients, including the amount of blood returned and the resting time after configuration.
3. Use questionnaires to evaluate patients during the infusion process, with a scale of 1–10, with 1 being very dissatisfied and 10 being very satisfied.
4. Regarding our experiments on the application of the IoT technology to the infusion management and control system, the nursing staff can freely evaluate it and can list the advantages and disadvantages and the problems that may arise during the implementation process.
5. In data collection method, nurses collect the number of infusion-related electric bells and the number of entering and exiting nurse stations. The daily steps of the nurse are automatically recorded via smartphones and WeChat applications. The nurse during the operation and the chief nurse recorded the number of blood drops that were dispensed for verification. The rest time after prescription refers to the difference between the use time of the signature of the nurse in charge and the time before the prescription is completed. The head nurse used the questionnaire after treatment to investigate the evaluation of patients' infusion management. In the nurse's assessment, the head nurse used the question form after the experiment to investigate the person in charge of the infusion monitoring system.
6. The SPSS22.0 statistical software was used for statistical data analysis. The measurement data was expressed as *x* ± *s*, and the comparison of the means between the two groups was made by *t*-test; the count data was expressed in %, and the comparison was made by *χ*2 test. *P* < 0.05 indicates statistical significance.

### 3.4. Experimental Process

Firstly, on the computer page of the nurse station, various data sent from the injection screen can be displayed, and the computer can decode the data for pumping. On the computer screen, each bed is represented by a rectangular box. The background of the infusion group is different. The color indicates various operating conditions of the screen, and the gray indicates that the screen is invalid. White means that the screen is active and the injection has not yet started. The blue liquid in the container is already at the bottom. If the yellow liquid flashes, it means that the first injection will try to end the quick warning, and the red flashing means that the second alarm will be triggered when the injection is about to end. Now the nurse must deal with that and either change the injection or stop the injection. If the rectangular background of the room is flashing red, it means that the data is sent incorrectly and you need to confirm the data receiver or network communication problem. If too much liquid is injected, there will be defects. Please confirm the reason before lying in bed and eliminate the error.

Secondary, you can display the information bar on one screen at the same time and inject the data of the entire screen. The internal structure of the screen uses an electronic gravity sensor, a low transmittance amplifier, an analog-to-digital converter, and a microprocessor. The nurse can connect through the console computer, use a special operating system driver to receive all the data sent, and decode and analyze the data. Nurses can collect various parameters related to injection and display them on the computer screen. Please be clear. After the infusion set is hung on the screen hook, the computer records the time when the infusion starts, and the monitor measures the total weight of the infusion bag and the infusion. According to the 500 ml microprocessor, the weight of 500 ml is automatically determined. After the injection starts, the liquid in the container gradually decreases. The microprocessor processes and analyzes the reduced value and the time to receive the injection speed and calculates the time required to inject the remaining liquid into the container according to the speed. After the injection is completed, an alarm signal will be issued. During the injection, the injection was interrupted. At this time, the injection speed is calculated as zero, and the screen immediately sends an injection failure message. Please let the nurse reminds you that the injections of the patients who must be dealt with within the time failed. The nurse can also see the flashing red pattern on the screen to deal with the time after bed.

## 4. Application Analysis of Infusion Control System Based on Internet of Things Technology in Joint Orthopedics Nursing Work

### 4.1. Comparison of Infusion Quality Indicators between the Internet of Things Infusion Control Group and the Control Group

The experimental subjects in this paper are divided into the conventional group and the IoT infusion management group. The comparison of the two infusion quality indicators is shown in Table 1. As can be seen from Table 1, *P* is all less than 0.05, indicating that the data are all statistically significant. In terms of infusion-related ringing rate indicators, the data of the IoT group are only about 30%, which is significantly lower than the ringing rate of the control group, indicating that the infusion management based on IoT technology has a good effect. And the accuracy rate of the drip count is significantly higher than the accuracy rate of the control group. The digital medical process can improve the medical situation very well.

It can be seen from Figure 3 that, in general, the infusion management and control system based on the Internet of Things technology has greatly improved various quality indicators compared to the conventional infusion.

### 4.2. Comparison of Work Efficiency between IoT Infusion Control Group and Control Group

The work efficiency of nurses can be measured from the number of steps walked, the round-trip time, the number of round trips, and other indicators. This article selects the above three indicators for testing. The test results are shown in Table 2.

It can be seen from Table 2 and Figure 4 that the efficiency of the IoT infusion management group is significantly higher than that of the control group. The round-trip time without purpose is only half of the control group, which greatly reduces unnecessary walking time and improves work efficiency; the number of round trips is 1/3 of the control group. In addition, the information collection time is 0. This is because the database of the Internet of Things can realize real-time upload and delivery of relevant information, without the need for nurses to manually collect information, which greatly saves ineffective working time. The nursing staff in the infusion management group of the Internet of Things took 10557.9 ± 600.6 steps per day on duty, and the number of steps taken by the nursing staff in the control group was 11385.9 ± 745.9. At the same time, the index *P* of the table is less than 0.05, which accords with the general significance in statistics and has experimental value.

### 4.3. Comparison of the Resting Time and Infusion Process Score between the Two Groups of Patients in the IoT Infusion Control Group and the Control Group

Table 3 shows the scoring table of the infusion process and the static time comparison table after liquid configuration of the IoT group and the control group. From Table 3 and Figure 5, it can be seen that the static time of the IoT group after liquid configuration is 4.9±0.95, while the control group's time was 12.1±1.3. The IoT infusion management group allowed patients to wait for an infusion significantly shorter than that of the conventional group, which effectively improved the infusion efficiency. During the infusion process, the IoT group got a score of 8.4±0.9, and the control group got a score of 6.6±0.9. There was a big difference between the two. The IoT management group received much more praise than the control group, and the score was significantly higher than the control group, which indicates that the IoT infusion control group is more likely to be favored by patients and has a better sense of infusion experience.

### 4.4. The Satisfaction of Patients in the IoT Infusion Group and the Control Group for Nursing Work

This paper implements two different types of infusion methods: one is based on the Internet of Things technology for infusion management and control, and the second is conventional personnel infusion management and control. From the four aspects of humanized service, infusion operation speed, whether to check during the infusion and the time to replace the infusion bottle and the patients' satisfaction with the infusion are considered and compared.

It can be seen from Table 4 and Figure 6 that there are big differences before and after the implementation of the IoT infusion control system. After the implementation, the humanized service has been more perfect, the operation time of fluid replacement and infusion has become shorter, there is no need for more inspection time during the infusion, and fluid replacement can be performed in the first time. This shows that, after the Internet of Things infusion management and control, in the process of joint orthopedics nursing, the work efficiency of nursing staff can be greatly improved, the duration of infusion work can be shortened, and the satisfaction of nursing services to patients can be improved.

During the injection, the needle often penetrates the blood vessel and fluid leaks into the subcutaneous tissue. If you change the direction of the needle or press the infusion tube with the patient's hands and feet, the injection failure and droplets will disappear. Therefore, the workload of the nurse inspection is very heavy. Patients and their families must always pay attention to the injection process. They cannot rest and have different medical risks. From the experimental results of this study, the infusion control system of the Internet of Things can clearly display the infusion situation of each patient, including infusion information, infusion time, and remaining infusion volume, so that medical staff can ensure the first-hand information to deal with different situations in time.

### 4.5. Comparison of Evaluation Indicators between the Two Groups

The research results in Table 5 show that, according to the routine, a short-time manual inspection requires one hour. Compared with the experimental group, the difference is statistically significant (*P* < 0.05). This may be caused by the inability of the previous manual monitoring methods to effectively monitor the injection. In order to ensure the safety of the infusion, nurses must check repeatedly to avoid the decrease of the infusion line after the patient's physique is changed or the patient's lack of compliance, adjust the rate of decline at will, and increase the burden on the nursing staff. The intelligent infusion monitoring system can automatically measure and analyze the data of the entire infusion process, and send the data to the terminal computer nurse station and portable real-time terminal. When an exception occurs, an automatic alarm is triggered. During the injection process, when the remaining liquid volume is 15 ml, the system can monitor the patient's remaining liquid volume according to defined parameters. The monitoring system issued an alarm for the first time. The software interface uses a fixed color to mark the alarm clone number and completes the response to the remaining liquid volume through voice commands. Liquid volume: when the remaining amount of liquid injected into the system wakes up again, the nurse will help understand the remaining amount of ml. Effective adjustment of injection engineering: from the perspective of infusion quality management, the infusion monitoring system based on the IoT recognizes the actual management of infusion and the progress and end of the infusion process from the very beginning. At the same time, retrospective management that reflects the wisdom and perfection of modern medical management can also be implemented, which helps to improve the quality of medical services and nursing business.

From Figure 7, we can see that the picture on the left is the picture of knee osteoarthritis, the picture on the right is the picture after the nursing of joint orthopedics, and the picture on the right is obviously normal, which indicates that the patients after the nursing of joint orthopedics have a better recovery, the recovery time is shorter, and the satisfaction of patients is higher.

## 5. Conclusion

This paper mainly studies the application of the infusion control system based on the IoT technology in joint orthopedics nursing work. Through in-depth research on the IoT technology, RFID technology, cloud computing technology, and so on, we fully learn from the experience of the past infusion system to build a brand new infusion management and control system based on IoT technology. In joint orthopedics nursing and treatment, it can play its role well, improve the efficiency of infusion, improve the current situation of infusion, and improve the satisfaction of patients.

The innovations of this paper are as follows: first, combining qualitative research with quantitative research, fully combining research data with practical application value, and showing the practical value of the research in this paper; second, combining theoretical research with empirical research and in-depth study based on the theoretical basis of the IoT technology combined with the actual infusion control system to conduct empirical investigations.

The research direction of this paper is that the application prospect and scope of the IoT technology in the medical and health field are very broad, and they will further promote the development of the IoT industry. However, there are still some technical problems in the research of this paper, such as the high cost of data compression algorithms, data security issues, high application costs, inconsistent technical standards, difficulty in protecting privacy, and weak competitiveness of service companies, which still restrict the development of the industry.

## Figures and Tables

**Figure 1:** Key technology roadmap of Internet of Things (IoT).

**Figure 2:** Composition chart of Internet infusion detection and control.

**Figure 3:** Comparison of infusion management quality indicators between the two groups.

**Figure 4:** Work efficiency of two groups of nursing staff (X±S).

**Figure 5:** Comparison of standing time and infusion process score between the two groups after liquid configuration.

**Figure 6:** Comparison of infusion satisfaction of patients before and after implementation of IoT technology.

**Figure 7:** X-ray manifestations of knee osteoarthritis and normal after nursing.

**Table 1:** Comparison of infusion management quality indicators between the two groups.

Group	N	Infusion-related ringing rate/%	Drop number accuracy/%	Infusion satisfaction rate/%
Internet of Things infusion management group	358	29.8	98.8	98.5
Control group	210	81.3	90.1	92.1
*χ* ^2^		18.91	29.64	12.65
P		0.001	0.001	0.001

**Table 2:** Work efficiency of two groups of nursing staff (X±S).

Group	Aimless round-trip time (t/min)	Number of round trips	Average daily steps	Information collection time (t/min)
IoT infusion management group (*N* = 358)	5.7±0.6	3.3±0.6	10557, 9 ± 600, 6	0
Control group (*N* = 210)	10.3±1.2	10.2±0.6	11385, 9 ± 745, 9	7.4±1.2
*χ* ^2^	9.29	24.12	15.78	17.82
*P*	0.001	0.001	0.001	0.001

**Table 3:** Comparison of standing time and infusion process score between the two groups after liquid configuration.

Group	*N*	Standing time after drug configuration (min)	Infusion process score
IoT group	358	4.9±0.95	8.4±0.9
Control group	210	12.1±1.3	6.6±0.9
t		18.32	6.31
P		0.000	0.000

**Table 4:** Comparison of infusion satisfaction of patients before and after implementation of IoT technology.

Time	Humanized service in place	Operating speed	There were inspections during the infusion period	Change the liquid in time
Before implementation	14.73±1.54	15.18±1.64	19.34±1.29	13.89±1.83
After implementation	19.76±1.37	19.95±1.86	13.16±1.48	19.76±1.38
X2	5.135	4.852	6.123	6.136
P	0.001	0.001	0.001	0.001

**Table 5:** Comparison of two groups of evaluation indexes.

Group	Number of cases	Detection accuracy of infusion residue (bag/bottle)	Observation and education time of nurses (min)	Patient satisfaction (grade)
IoT group	358	5.38±1.23	149.97±12.17	55.97±1.89
Control group	210	2.23±0.88	118.03±9.65	52.56±2.24
T value		25.935	25.424	15.112
*P*		<0.001	<0.001	<0.001

## Data Availability

No data were used to support this study.
